# Phytochemical, Antioxidant, Antihyaluronidase, Antityrosinase, and Antimicrobial Properties of *Nicotiana tabacum* L. Leaf Extracts

**DOI:** 10.1155/2022/5761764

**Published:** 2022-08-29

**Authors:** Adchara Prommaban, Kantaporn Kheawfu, Chuda Chittasupho, Sasithorn Sirilun, Kirachuda Hemsuwimon, Wantida Chaiyana

**Affiliations:** ^1^Department of Pharmaceutical Sciences, Faculty of Pharmacy, Chiang Mai University, Chiang Mai 50200, Thailand; ^2^Research Center of Pharmaceutical Nanotechnology, Chiang Mai University, Chiang Mai 50200, Thailand; ^3^Innovation Center for Holistic Health, Nutraceuticals, and Cosmeceuticals, Faculty of Pharmacy, Chiang Mai University, Chiang Mai 50200, Thailand; ^4^Tobacco Authority of Thailand, Leaf Department, Maejo Tobacco Experiment Station, Chiang Mai 50290, Thailand

## Abstract

*Nicotiana tabacum* L. (tobacco) is an important and valuable crop for the cigarette industry. However, cigarette cessation has been encouraged worldwide. Therefore, this study aimed to investigate the potential of *N. tabacum* leaf extract use in other industries besides cigarette production, especially cosmeceutical industries, which are of interest for increasing the value and widening the applications of *N. tabacum*. The leaves of *N. tabacum* var. Virginia and Turkish were extracted by maceration using 95% v/v ethanol or petroleum ether. The extracts were evaluated for their phytochemical compositions, antioxidant capacity, and anti-aging, antimelanogenic, and antimicrobial activities. The phytochemical screening of the extracts revealed terpenoids, steroids, alkaloids, tannins, and carbohydrates in all of the *N. tabacum* leaf extracts. The total phenolic content was detected to be the highest in the ethanolic extract of Virginia tobacco leaf, which had the most significantly potent antioxidant and antihyaluronidase activity (*P* < 0.05). On the contrary, the extracts from the Turkish variety demonstrated the most powerful antimicrobial activity against *Staphylococcus aureus*. Thus, ethanolic extracts of *N. tabacum* var. Virginia are suggested as good natural anti-aging ingredients with potent antioxidant and antihyaluronidase effects, whereas the leaf of *N. tabacum* var. Turkish is suggested as a good source of natural antimicrobial components, particularly for *S. aureus* inhibition. In summary, in addition to the cigarette industry, *N. tabacum* leaf could be a source of pharmaceutical and cosmeceutical compounds, particularly natural anti-aging and antimicrobial ingredients.

## 1. Introduction

*Nicotiana tabacum* L., or tobacco, is a member of the Solanaceae family. It is one of the most commercially valuable agricultural crops in the world and is usually used in the cigarette industry. In Thailand, *N. tabacum* is grown in the northern and northeastern regions, and is also used as a raw material for the manufacture of cigarettes. Although cigarettes have adverse effects on humans and the environment, *N. tabacum* contains several useful phytochemical components that could be applied in other industries. *N. tabacum* has been reported to contain large numbers of secondary metabolites exerting many biological and pharmacological activities [1, 2]. For example, previous research found that alkaloids derived from plant extracts had an anti-insect effect, which is important in agriculture, as well as exerting health benefits for Alzheimer's and Parkinson's diseases [3–5]. In addition, solanesol and its derivatives have antibacterial, anticancer, anti-inflammatory, and antioxidant properties [6]. Its polyphenols also presented antioxidant capacity, along with playing an important role in the prevention of various diseases, such as hyperlipidemia, arthrosclerosis, cardiovascular disease, and cancer [7, 8]. Moreover, the phenolic acids, particularly chlorogenic acid and rutin, contributed to the potential for both antioxidant and antimicrobial activities [9]. Overall, extracts of *N. tabacum* show the presence of abundant bioactive molecules that can provide many health benefits in humans. Apart from the pharmaceutical industries, the cosmeceutical industries are also an interesting market that could promote the value of natural resources. Since *N. tabacum* has been reported to display various pharmaceutical effects, it could be applied in the cosmeceutical industries. Regarding the various biological functions of *N. tabacum*, different parts of the plant have been examined. A variety of phytochemical components have been found in various parts of *N. tabacum*, resulting in numerous biological activities. Antimicrobial activity has been detected in the leaves, stems, and roots [10–14]. Similarly, antioxidant activities were also found in various parts of *N. tabacum*, including the leaves, roots, and stems [13, 15, 16]. According to the mentioned properties, *N. tabacum* has the potential to be used as an active ingredient in pharmaceutics and cosmetics, leading to the greatly increased value of this plant. However, the leaves are easier to utilize than the roots and stems since the plant does not need to be uprooted or exterminated.

Among several varieties of *N. tabacum*, the Virginia and Turkish varieties are widely cultivated in the northern regions of Thailand. Therefore, our research team was interested in evaluating the phytochemical components and their biological and pharmacological activities, including antioxidant, anti-aging, whitening, and antimicrobial effects, of *N. tabacum* var. Virginia and Turkish leaf extracts. Since there was no previous study on the anti-aging and antimelanogenic properties of *N. tabacum* extract, the goal of this research was to investigate the potential of tobacco for use in cosmeceuticals for the further development of tobacco-based cosmeceutical products.

## 2. Materials and Methods

### 2.1. Plant Material

Fresh leaves of *N. tabacum* var. Virginia and Turkish were identified and authenticated by Miss Wannaree Charoensup, a specialized botanist at the Herbarium of Faculty of Pharmacy, Chiang Mai University, and Mrs. Kirachuda Hemsuwimon, an agricultural specialist of Tobacco Authority of Thailand, Leaf Department, Maejo Tobacco Experiment Station, Chiang Mai, and locally obtained from the Maejo Tobacco Experiment Station, Chiang Mai, Thailand, under the Tobacco Authority of Thailand (TOAT), in May 2021. Voucher specimen No. 0023300 of *N. tabacum* var. Virginia and No. 0023301 of *N. tabacum* var. Turkish were deposited at the Herbarium of the Faculty of Pharmacy, Chiang Mai University.

### 2.2. Chemical Reagents

2,2′-Azinobis 3-ethylbenzothiazoline-6-sulphonate (ABTS), 2,2-diphenyl-1-picrylhydrazyl-hydrate (DPPH), 2,4,6-tripyridyl-s-triazine (TPTZ), 6-hydroxy-2,5,7,8-tetramethyl chroman-2-carboxylic acid (Trolox), ammonium thiocyanate (NH_4_SCN), ferrous chloride (FeCl_2_), kojic acid, L-tyrosine, linoleic acid, oleanolic acid, ferrous sulfate (FeSO4), potassium persulfate (K_2_S_2_O_8_), sodium acetate trihydrate (CH_3_COONa.3H_2_O), sodium chloride (NaCl), sodium sulfate anhydrous (Na_2_SO_4_), and tyrosinase from mushroom (EC 1.14.18.1) were purchased from Sigma-Aldrich (St. Louis, MO, USA). Acetic acid, hydrochloric acid, ethanol, calcium chloride (CaCl_2_), chloroform, de-ionized (DI) water, dimethyl sulfoxide (DMSO), glacial acetic acid, petroleum ether, and sulfuric acid (H_2_SO_4_) were purchased from RCI Labscan Co., Ltd. (Bangkok, Thailand).

### 2.3. Plant Extraction

Fresh leaves of *N. tabacum* var. Virginia and Turkish were washed and dried. The leaves of *N. tabacum* var. Virginia were dried at a temperature of 32–75°C for 6 days, whereas those of var. Turkish were dried at a temperature of 25–30°C for 20 days. The dried leaves were cut into the smallest pieces possible and divided into two portions to be macerated with ethanol and petroleum ether for 48 h. All the leaves were removed from solvents, filtered with Whatman No. 1, and evaporated in a rotary evaporator (EYELA N-N series, Labfirst Scientific Instruments (Shanghai) Co., Ltd., Shanghai, China). Each residue was collected and its extraction yield calculated.

### 2.4. Chemical Composition Determination

#### 2.4.1. Phytochemical Screening

Preliminary phytochemical screening of *N. tabacum* leaf extracts was performed to evaluate the quantities of carbohydrates, glycosides, terpenoids, steroids, alkaloids, tannins, and anthraquinones. Carbohydrates were evaluated using Molisch and Benedict's test [17]. Glycosides were evaluated by the Keller–Kiliani test [18]. Terpenoids were evaluated by the Salkowski test [18]. Steroids were evaluated by the Liebermann–Burchard test [19]. Alkaloids were evaluated using different reagents, including Dragendorff's, Mayer's, Wagner's, and Hager's reagents [20, 21]. All the experiments were carried out in triplicate. Tannins were evaluated using different reagents, including 0.5% gelatin, 1% quinine sulfate, 1% lead acetate, and vanillin reagents [21–23]. Anthraquinones were evaluated using Borntrager's test [23]. All the experiments were carried out in triplicate.

#### 2.4.2. Total Phenolic Content

The Folin–Ciocalteu method was used to determine the total phenolic content of *N. tabacum* extracts [24]. The reaction mixture consisted of 20 *μ*l of extract, 80 *μ*l of freshly prepared Folin–Ciocalteu reagent, and 100 *μ*l of 7.5% sodium carbonate, which were then incubated at room temperature and in the dark for 2 h. The mixture was measured for absorbance at 765 nm, and we calculated the phenolic content using gallic acid as a standard; results were expressed as gallic acid equivalents (GAE). Three independent experiments, repeated in triplicate, were performed.

#### 2.4.3. Determination of Nicotine Content Using High-Performance Liquid Chromatography (HPLC)

The identification of nicotine in *N. tabacum* extracts was performed via the high-performance liquid chromatography (HPLC) method (Hewlett-Packard, Inc., Palo Alto, CA, USA). A C-18 reverse phase column (Hypersil ODS, 4.6 × 150 mm, Agilent Technologies, Inc., CA, USA) was used to evaluate the nicotine content. The mobile phases consisted of solvent *A* containing sodium acetate: methanol: triethylamine in a ratio of 88 : 12 : 0.5 (v/v) and solvent *B* containing methanol with a flow rate of 1 mL/min. The samples (5 *μ*l) were injected and separated in peak areas for 30 min, and then detected with an UV detector at a wavelength of 259 nm. Peak areas of the eluted compounds were recorded and integrated with the HPLC software. Persisting nicotine compounds were identified by comparison with nicotine standard [25]. All experiments were carried out in triplicate.

### 2.5. Antioxidant Activity Determination

#### 2.5.1. DPPH Assay

The radical scavenging activity of *N. tabacum* extracts against DPPH radicals (DPPH•) was assessed using the method established by Chaiyana et al. [24]. The reaction mixture contained 20 *μ*L extract and 180 *μ*L of 167 *μ*M DPPH solution, incubated in dark conditions at ambient temperature for 30 min, and measured at absorbance of 520 nm (Microplate Reader EZ Read 2000, Biochrom Ltd., Cambridge, UK). Three independent experiments, repeated in triplicate, were performed. The percentage of DPPH inhibition was computed using the following calculation: % DPPH inhibition = [(*A* − *B*)/*A*] × 100, where *A* is the absorbance of the control, and *B* is the absorbance of the sample.

#### 2.5.2. ABTS Assay

The radical scavenging activity of *N. tabacum* extracts against ABTS cationic radicals (ABTS^•+^) was assessed using the method described by Laosirisathian et al. [26]. ABTS^•+^ was produced by combining 2 mL of 7 mM ABTS and 3 mL of 2.45 mM potassium persulfate oxidant under 16–24 h incubation, in dark conditions, at ambient temperature. The working solution was prepared by diluting ABTS^•+^ with ethanol until the OD reached 0.7 ± 0.1 at 750 nm. For the scavenging reaction, 20 *μ*L of sample was mixed with 180 *μ*L of ABTS^•+^ solution, incubated in dark conditions at ambient temperature for 5 min, and measured at absorbance of 750 nm (Microplate Reader EZ Read 2000, Biochrom Ltd., Cambridge, UK). The results were demonstrated in terms of Trolox equivalent antioxidant capacity (TEAC). Three independent experiments, repeated in triplicate, were performed.

#### 2.5.3. Ferric Reducing Antioxidant Power (FRAP) Assay

The FRAP of *N. tabacum* extracts was determined by following previous studies by Saeio et al. and Chaiyana et al. [24, 27]. For FRAP reagent preparation, 0.3 M acetate buffer (pH 3.6), 0.01 M 2,4,6-tripyridyl-s-triazine (TPTZ) in 0.04 M HCl, and 0.02 M FeCl_3_ were combined in proportions of 10 : 1 : 1. The reaction mixture contained 20 *μ*L of extract and 180 *μ*L of FRAP reagent, incubated in the dark at ambient temperature for 5 min, and measured at absorbance of 595 nm (Microplate Reader EZ Read 2000, Biochrom Ltd., Cambridge, UK). The results were recorded in terms of equivalent capacity (EC_1_) when compared to the ferric sulfate (FeSO_4_) standard curve. Three independent experiments, repeated in triplicate, were performed.

#### 2.5.4. Ferric Thiocyanate Assay

The lipid peroxidation inhibition of *N. tabacum* extracts was determined by the ferric thiocyanate (FTC) method, following the method of Chaiyana et al. [24]. The reaction mixture contained 50 *μ*L of extract, 50 *μ*L of 50% w/v linoleic acid diluted in DMSO, 50 *μ*L of 10% w/v of ammonium thiocyanate (NH_4_SCN), and 50 *μ*L of 2 mM ferrous chloride (FeCl_2_), incubated at 37°C for 1 h, and measured at absorbance of 500 nm (Microplate Reader EZ Read 2000, Biochrom Ltd., Cambridge, UK). Three independent experiments, repeated in triplicate, were performed. The percentage of lipid peroxidation inhibition was computed using the following calculation: % Lipid peroxidation inhibition = [(*A* − *B*)/*A*] × 100, where *A* is the absorbance of the control, and *B* is the absorbance of the sample.

### 2.6. Antihyaluronidase Activity Determination

The antihyaluronidase activity of *N. tabacum* extracts was evaluated following the method of Chaiyana et al. [28]. The reaction mixture consisted of 20 *μ*L of extract and 100 *μ*L of 15 U/mL hyaluronidase solution, which was then incubated at 37°C for 10 min. The incubated mixtures were combined with 0.1 mL of 0.03% w/v hyaluronic acid dissolved in 0.02 M phosphate buffer (pH 5.35), which was then incubated at 37°C for 45 min. After incubation, 1 mL of 0.1% w/v bovine serum albumin was added, and the mixture was incubated at room temperature for 10 min and measured at absorbance of 600 nm (Microplate Reader EZ Read 2000, Biochrom Ltd., Cambridge, UK). Three independent experiments, repeated in triplicate, were performed. The percentage of hyaluronidase inhibition was computed using the following calculation: % Hyaluronidase inhibition = [(*A* − B)/A] × 100, where *A* is the absorbance of the control, and *B* is the absorbance of the sample.

### 2.7. Antityrosinase Activity Determination

The antityrosinase activity of *N. tabacum* extracts was assessed following the method established by Prommaban et al. [29]. The reaction mixture contained 10 *μ*L of extract and 30 *μ*L of tyrosinase, incubated at room temperature for 10 min. Then, the mixtures were combined with 0.1 mL of substrate and 2.5 mM of L-tyrosine or L-DOPA, incubated at room temperature for 30 min, and measured at absorbance of 450 nm (Microplate Reader EZ Read 2000, Biochrom Ltd., Cambridge, UK). Three independent experiments, repeated in triplicate, were performed. The percentage of tyrosinase inhibition was computed using the following calculation: % Tyrosinase inhibition = [(*A* − *B*)/*A*] × 100, where *A* is the absorbance of the control, and *B* is the absorbance of the sample.

### 2.8. Antimicrobial Activity Determination

The antimicrobial activity of *N. tabacum* extracts was examined against 4 reference bacterial strains obtained from the American Type Culture Collection (ATCC): *Staphylococcus aureus* (ATCC25923), *Staphylococcus epidermidis* (ATCC12228), *Propionibacterium acnes* (ATCC6919), and *Pseudomonas aeruginosa* (ATCC27853). Antimicrobial assays were performed using the agar disc diffusion, minimum inhibitory concentration (MIC), and minimum bactericidal concentration (MBC) techniques by following previously established methods.

#### 2.8.1. Agar Disc Diffusion Method

The bacterial inoculum was diluted in phosphate-buffered saline (pH 7.4) to obtain turbidity visually comparable to the McFarland N° 0.5 standard (1 × 107 CFU/mL). Each inoculum was spread over tryptic soy agar (TSA) plates. For disc preparation, 10 *μ*l of each extract was dropped onto a 5 mm diameter paper disc and then plated on a TSA plate containing bacteria, and incubated at 37°C for 24 h. Reference antibiotics used in this study were 25 *μ*g of Ampicillin® and Penicillin®. The inhibitory zones around the discs were observed, measured, and expressed in mm [30]. All the experiments were carried out in triplicate.

#### 2.8.2. Minimum Inhibitory Concentration (MIC) Method

MIC was characterized by the lowest concentration that inhibited the visible bacterial growth. Briefly, Mueller–Hinton Broth (MHB) was plated in a 96-well plate, and then, the extracts were twofold diluted in MHB at a ratio of 1 : 2 to 1 : 64. The bacteria were added to test wells with a final concentration of 1 × 10^5^ CFU/mL and incubated in 37°C for 24 h. The growth of bacteria was observed; a clear solution indicated no growth, and a turbid cloudy solution indicated bacterial growth [31]. All experiments were carried out in triplicate.

#### 2.8.3. Minimum Bactericidal Concentration (MBC) Method

The concentration presenting no growth visible in MIC was used to test the MBC. The same concentration of MHB, along with the extracts, was spread over Mueller–Hinton agar (MHA) plates and then incubated at 37°C for 24 h. The growth of bacteria was observed and reported as the bactericidal concentration [31]. All experiments were carried out in triplicate.

### 2.9. Statistical Analysis

All experimental data were expressed as mean ± SD. Statistical data were analyzed using Tukey's post hoc test and one-way analysis of variance (ANOVA) in GraphPad Prism (version 8.0; GraphPad Software). Statistically significant differences were demonstrated when *P* < 0.05.

## 3. Results and Discussion

### 3.1. Yield of *N*. *tabacum* Extracts

Different varieties and solvent extractions of *N. tabacum* leaves are presented as percent yields according to Table 1. The ethanolic extracts from both *N. tabacum* varieties (VL-E and TL-E) exhibited higher percent yields than those obtained with petroleum ether extraction (VL-P and TL-P). This could indicate that *N. tabacum* extracts contain both nonpolar and polar compounds, but they were composed of huge amounts of polar compounds, which can be extracted with a polar solvent such as ethanol. However, there were no differences in the amount of yield between the two varieties in ethanolic extraction, but *N. tabacum* var. Turkish had a slightly higher yield than Virginia during part of the petroleum ether extraction process.

### 3.2. Chemical Constituents of *N*. *tabacum* Extracts

Preliminary phytochemical screening of *N. tabacum* extracts was performed to detect carbohydrates, glycosides, terpenoids, steroids, alkaloids, tannins, and anthraquinones, with the results provided in Table 2. Some phytochemical compounds—terpenoids, steroids, alkaloids, and tannins—were found in all extracts, but only carbohydrates were found in the ethanolic extracts of both varieties. Interestingly, steroids were more abundant in Turkish than in Virginia varieties. However, glycosides and anthraquinones were not detected in the extracts. As is known, the phytochemical composition of a plant demonstrates its various pharmacological and health benefits. Terpenoids are secondary metabolites found in many plants and widely used for flavoring and fragrance in the food and pharmaceutical industries [8]. Alkaloids display various biological properties, such as anti-inflammatory, antioxidant, antibacterial, and anticancer activities [8, 32]. Steroids show anti-inflammatory, anticancer, antioxidant, and anti-atherogenicity activities [33]. Tannins, a component of natural polyphenols, are widely used in medical applications, including as anti-inflammatory and diuretic agents against stomach and duodenal tumors [34]. This investigation presented some phytochemical compounds similar to the reports of Peter et al. and Kaushik et al. [21, 35], who also determined the compounds in extracts of *N. tabacum* leaves. In addition to the carbohydrates, alkaloids, phenolic compounds, tannins, flavonoids, steroids, and terpenoids reported in the current study, Peter et al. revealed the presence of resins and essential oil in the *N. tabacum* leaves [21], whereas Kaushik et al. revealed the presence of saponins and terpenes [35]. Moreover, different parts of *N. tabacum*, such as the root and stem, yield slightly different phytochemical compounds from the leaves [13, 36]. Sharma et al. revealed the presence of only flavonoids, alkaloids, and saponins in the stems of *N. tabacum*, whereas no carbohydrates, polyphenols, tannins, steroids, or terpenoids were detected [13]. On the contrary, Sunil et al. revealed the presence of flavonoids, phytosterols, triterpenoids, and tannins in the roots of *N. tabacum* [36]. In brief, variations in phytochemical composition could depend on the plant parts, varieties, solvents, and methods of extraction.

Phenolic compounds from plants display a variety of biological functions, especially as antioxidant agents with high reactive oxygen species (ROS) radical scavenging capacity. In this study, the total phenolic content of *N. tabacum* extracts was calculated using a gallic acid calibration curve and represented as gallic acid equivalents (GAE) per gram dry extract weight. According to Table 3, ethanolic extracts of both *N. tabacum* varieties had higher total phenolic content than petroleum ether extracts. VL-E showed significantly higher amounts than TL-E, TL-P, and VL-P. These results could imply that the polarity of the solvent used in extraction influences the concentrations of phenolic compounds in plant extracts. Because phenols are highly soluble in polar solvents, they can provide higher concentrations of phenols than nonpolar solvents [37]. The amounts of phenolics found in ethanolic extracts in this study were significantly higher than previously reported by Zou et al., who reported that the methanolic extract of *N. tabatum* had the highest amount in terms of total phenolic content, at 24.82 ± 0.07 mg GAE/g extract [38]. However, different solvents and extraction methods were considered. Moreover, Soumeya et al. found that the leaf extract has higher amounts of phenols than the other parts of *N. tabacum* [39], which could indicate that *N. tabacum* leaf extracts might contain a large number of phenolic compounds that exert antioxidant and other biological properties.

Nicotine is a major and common alkaloid that is generated by ornithine metabolism [40]. It is frequently found in *N. tabacum* or tobacco and is accumulated in tobacco leaves. Despite the fact that nicotine in tobacco causes disease and death in a large number of people, a mild, safe degree of purified nicotine exhibits potential medical uses—for instance, in the reduction of body weight, reduction of stress, and protection against some diseases [41]. The HPLC fingerprint of the nicotine compound presented a retention time of approximately 4.5 min (Figure 1(a)). Nicotine compound was found in VL-E and VL-P extracts and expressed as 5.27 ± 0.13% and 1.01 ± 0.16%, respectively (Figures 1(b) and 1(c)). Nonetheless, no peak area for the nicotine compound was found in TL-E and TL-P extracts. It is possible that nicotine content varies according to the *N. tabacum* variety. The results were well in line with the previous work from Ghaleb et al., who found that the dry weight of N. tabacum var. Virginia leaf extract expressed nicotine in an amount of 6.7% and an even lower amount was detected in other species such as Burlip, Kstrina, and Zegrin [42]. These results indicated that *N. tabacum* var. Virginia contained higher nicotine content than other varieties, supporting our investigation. Another report also found that the concentrations of nicotine in samples in Bangladesh were in the relative range of 0.9 to 3.6% dry weight [43], representing a slightly lower amount than in our study. Moreover, the research by Mirjana and Kelly reported that several cultivated varieties of *N. tabacum* presented alkaloid content in the range of 0.17 to 4.93%. It was implied that the variation in the alkaloid content depended on the type, the process of tobacco production, and product development, resulting in a variety of nicotine concentrations [44].

### 3.3. Antioxidant Activities of *N*. *tabacum* Extracts

Regarding chemical composition properties, several methods were used for determining the antioxidant activity of *N. tabacum* extracts. The antioxidant activities of the extracts are shown in Figure 2. At the same concentration of the extracts, ethanolic extracts, especially VL-E, exerted potent antioxidant power, with significantly decreased radicals for both DPPH and ABTS, as well as significantly potent ferric reducing power (*P* < 0.05). It could be suggested that the phenolic compounds of *N. tabacum* extracts were responsible for its potent antioxidant effects, since VL-E contained the significantly highest total phenolic content. On the contrary, petroleum ether extracts, TL-P and VL-P, inhibited lipid peroxidase more significantly than ethanolic extracts. This could be due to nonpolar extracts facilitating a large decrease in lipid peroxidase activity. However, the inhibitory activity against lipid peroxidase was only observed at a low level (below 20% inhibition).

Previous research focused on *N. tabacum* leaf extract, which was relevant to the present study. Wang et al. reported that ethanolic-extracted polyphenols from tobacco leaf possessed strong antioxidant activity when measured for the radical scavenging and lipid peroxidation inhibition activity [14]. Similarly, a previous investigation revealed that *N. tabacum* extracts exhibited strong antioxidant activities, including radical scavenging activity against DPPH and ABTS, as well as ferric reducing power, due to their polyphenols [38]. With regard to different methods to evaluate the antioxidant activity of tobacco, it was found that tobacco presented antioxidant capacity in the range of 66 to 230 *μ*mol Trolox equivalent/g dry weight using the ORAC method [45]. Furthermore, there was some evidence of antioxidant activity observed in various parts of *N. tabacum*, such as roots, stems, and flowers. According to a previous study by Al Lahham et al., *n*-hexane-extracted *N. tabacum* root extract showed the most potent antioxidant power, which was measured by the DPPH assay [9]. In addition, *N. tabacum* stem extract was found to contain important antioxidant enzymes such as superoxide dismutase and glutathione transferase, which also enhance the antioxidant activity [13]. Therefore, our study and the published literature indicate that polyphenols from tobacco plants exert antioxidant power.

### 3.4. Antihyaluronidase Activity of *N*. *tabacum* Extracts

Hyaluronic acid, or hyaluronan, is an important component of skin that is found in the epidermis and dermis. The function of hyaluronic acid is the maintenance of skin hydration and tissue homeostasis. Hyaluronic acid can be degraded by the hyaluronidase enzyme, resulting in small fragments, associated with loss of skin moisture and the subsequent induction of skin aging [46]. Recently, an alternative bioactive compound from plants was demonstrated as a potential ingredient in anti-aging agents. Several studies have investigated the anti-aging activities involving anti hyaluronidase activity in plant extracts [47, 48]. In a recent study, the inhibition of hyaluronidase activity achieved by *N. tabacum* extracts was assessed, as shown in Figure 3. Hyaluronidase activity was significantly inhibited by TL-E (29.5 ± 0.4% inhibition), similar to the effect of oleanolic acid (OA) (34.1 ± 1.3% inhibition), which is a reference standard for anti-aging activity. Moreover, VL-E and TL-P also strongly inhibited hyaluronidase activity, with 24.5 ± 6.4 and 20.9 ± 5.3% inhibition, respectively. The antihyaluronidase activity of *N. tabacum* extracts has not been reported to date. However, some previous studies reported that plant extracts containing polyphenols had a strong capacity for hyaluronidase inhibition [49, 50]. Therefore, plant extracts rich in phenolic compounds, including *N. tabacum* extracts, could enhance antihyaluronidase activity.

### 3.5. Antityrosinase Activity of *N*. *tabacum* Extracts

Melanogenesis is a biosynthetic pathway for the formation of the pigment melanin in human skin. Tyrosinase is a key enzyme in this process, as it converts L-tyrosine to L-DOPA, which is then oxidized to DOPA-quinone, and eventually synthesizes the melanin pigment [51]. In this regard, tyrosinase inhibitors are considered for skin whitening agents, which are important for the cosmetic industry. Therefore, various plant extracts have been tested as pharmaceuticals and cosmetics to prevent excessive melanin production in human skin. Despite the lack of previous research on *N. tabacum*'s antityrosinase activities, the presence of polyphenols, terpenoids, steroids, alkaloids, and tannins in the leaf extract suggests that *N. tabacum* has antityrosinase activities. A previous study revealed that several families of compounds contain molecules with antityrosinase properties, including phenols, polyphenols, steroids, and triterpenoids [52]. In this study, the inhibition of tyrosinase activity of *N. tabacum* extracts was assessed, as demonstrated in Figure 4. Kojic acid (KA) was used as a reference standard and exerted the highest tyrosinase inhibition (96.7 ± 0.5% inhibition). Meanwhile, VL-E and TL-E slightly reduced the tyrosinase activity. Several natural plant products have previously been described to attenuate the enzymatic activity involved in the melanogenesis process [53, 54]. Researchers suggested that plant extracts rich in bioactive compounds such as polyphenols and flavonoids, along with potent antioxidant properties, were correlated with the inhibition of tyrosinase enzyme activity [53]. This could suggest that the ethanol extracts of both varieties of *N. tabacum*, containing abundant phenolic compounds, support their capacity for tyrosinase inhibition.

### 3.6. Antimicrobial Activities of *N*. *tabacum* Extracts

The effects of N. tabacum extracts against bacteria were assessed, as shown in Tables 4–6. According to the agar disc diffusion method, all extracts inhibited the growth of *S*. *aureus*, *S*. *epidermidis*, *P*. *acnes*, and *P. aeruginosa* with different inhibition zones. TL-E and TL-P were most effective against *S*. *aureus*, while VL-E and VL-P were most effective for *P*. *acnes*. On the contrary, VL-P and TL-E reduced *S*. *epidermidis* and *P. aeruginosa* growth (Table 4). The standard antibiotics, Penicillin and Ampicillin, exhibited the largest inhibition zones, respectively. These results indicate that all extracts inhibited various bacteria involved in human skin. The susceptibility of bacteria depended on the *N*. *tabacum* varieties and solvent extraction method.

Tables 5 and 6 show the MIC and MBC values of *N. tabacum* extracts against the tested bacterial strains. TL-P and TL-E exhibited the most susceptibility to *S. aureus*, which was presented in ≥15.62 and ≥31.25 *μ*g/mL of extracts, respectively, in both MIC and MBC tests. In addition, the antibiotics, Ampicillin and Penicillin, revealed the lowest concentrations required to inhibit bacterial growth in all strains. Nevertheless, the other bacterial strains were susceptible to higher concentrations of all the extracts in the range of ≥125 to ≥500 *μ*g/mL. It could be concluded that the Turkish leaf extracts, TL-E and TL-P, were found to be effective antimicrobial agents against *S. aureus*.

Nowadays, researchers use extracts of plants for their pharmacological activities and antimicrobial activities. Several phytochemical compounds in tobacco plants, including polyphenols, terpenes, and polysaccharides, also exert antimicrobial activities [2]. Tandon and coworkers reported that the methanolic extract of *N. tabacum* leaf exhibited remarkable antimicrobial activity against *S. aureus* and *E. coli* [55]. Moreover, Akinpelu and Obuotor discovered that *N. tabacum* leaf extracts inhibited both Gram-positive and Gram-negative bacterial growth, such as *B. subtilis*, *P. aeruginosa*, and *S. aureus* [56]. In addition, previous studies indicated that the Nicotiana plant could be used as an effective antimicrobial agent [11, 14]. The investigation of the polyphenols extracted from tobacco leaf revealed high antioxidant and antimicrobial activity against *S. aureus* (17.66 ± 0.86 mm inhibition zone) [14] that was consistent with our findings. As previously reported, four types of bacteria caused skin infection and opportunistic infection in human skin. According to these results, *N. tabacum* var. Turkish (TL-E and TL-P) displayed a high percentage of inhibition and low concentrations of extracts in MIC and MBC tests, and it could be used to treat bacteria, especially *S. aureus*.

## 4. Conclusions

*N. tabacum* leaf extracts are enriched with various important phytochemical components, including alkaloids, terpenoids, steroids, and polyphenols. Ethanolic extracts of *N. tabacum* presented higher amounts of total phenolic compounds than petroleum ether extracts. The major alkaloid in tobacco, nicotine, was found in only the Virginia variety, and could not be observed in the Turkish one. The different types and amounts of phytochemical components depended on the varieties and solvent extraction methods. According to their polyphenols, both varieties also exhibited potent antioxidant and antihyaluronidase activities. Interestingly, the ethanolic extracts displayed excellent effects, especially VL-E. On the contrary, the extracts from the Turkish variety (both TL-E and TL-P) demonstrated the most powerful antimicrobial activity against *S. aureus*. Therefore, it could be suggested that the ethanolic extracts of *N. tabacum* var. Virginia are good natural anti-aging ingredients with potent antioxidant and antihyaluronidase effects, whereas the leaf of *N. tabacum* var. Turkish is suggested as a good source of natural antimicrobial compounds, especially for *S. aureus* inhibition. In brief, besides the cigarette industry, *N. tabacum* leaf would be a potential source of pharmaceutical and cosmeceutical ingredients. However, the principal component analysis was proposed for additional research. Besides, the safety of *N. tabacum* extracts should be assessed in a further study, in terms of both the cytotoxicity and the irritation potential.

## Figures and Tables

**Figure 1:** Chromatogram of nicotine standard (a) and *N. tabacum* extracts (VL-E, Virginia leaf ethanolic extract (b); VL-P, Virginia leaf petroleum ether extract (c)).

**Figure 2:** Antioxidant activities of *N. tabacum* extracts (VL-E, Virginia leaf ethanolic extract; VL-P, Virginia leaf petroleum ether extract; TL-E, Turkish leaf ethanolic extract; TL-P, Turkish leaf petroleum ether extract), ascorbic acid (AS), and Trolox. DPPH scavenging activities (a), ABTS scavenging activities (b), ferric reducing antioxidant power (c), and lipid peroxidation inhibition (d). The letters *a*, *b*, *c*, *d*, and *e* indicate significant differences among samples in each experiment, *P* < 0.05.

**Figure 3:** Antihyaluronidase activity of *N. tabacum* extracts (VL-E, Virginia leaf ethanolic extract; VL-P, Virginia leaf petroleum ether extract; TL-E, Turkish leaf ethanolic extract; TL-P, Turkish leaf petroleum ether extract) and oleanolic acid (OA). The letters *a* and *b* indicate significant differences among samples in each experiment, *P* < 0.05.

**Figure 4:** Antityrosinase activity of *N. tabacum* extracts (VL-E, Virginia leaf ethanolic extract; VL-P, Virginia leaf petroleum ether extract; TL-E, Turkish leaf ethanolic extract; TL-P, Turkish leaf petroleum ether extract) and kojic acid (KA). The letters *a*, *b*, and *c* indicate significant differences among samples in each experiment, *P* < 0.05.

**Table 1:** Yield of *Nicotiana tabacum* extracts.

Extracts	Yield (% w/w)
VL-E	12.80
VL-P	1.55
TL-E	12.33
TL-P	2.83

*Note.* TL-E, Turkish leaf ethanolic extract; TL-P, Turkish leaf petroleum ether extract; VL-E, Virginia leaf ethanolic extract; VL-P, Virginia leaf petroleum ether extract; w/w, weight by weight.

**Table 2:** Phytochemical screening of *N. tabacum* extracts.

Chemical constituents	Tests	Samples			
		VL-E	VL-P	TL-E	TL-P
Carbohydrates	Molisch's test	++	−	++	−
	Benedict's test	+	−	+	−

Glycosides	Keller–Kiliani test	−	−	−	−

Terpenoids	Salkowski's test	+	+	+	+

Steroids	Liebermann's test	+	+	++	++

Alkaloids	Dragendorff's reagent	+	+	+	+
	Mayer's reagent	+	+	+	+
	Wagner reagent	+	+	+	+
	Hager's reagent	+	+	+	+

Tannins	FeCl3 test solution	+	−	+	−
	0.5% gelatin test solution	+	+	+	+
	1% quinine sulfate test solution	+	+	+	+
	1% lead acetate	+	+	+	+
	Vanillin reagent	+	+	+	+

Anthraquinones	Borntrager's reagent	−	−	−	−

*Note*. ++, strong positive; +, positive; −, negative; TL-E, Turkish leaf ethanolic extract; TL-P, Turkish leaf petroleum ether extract; VL-E, Virginia leaf ethanolic extract; VL-P, Virginia leaf petroleum ether extract; w/w, weight by weight.

**Table 3:** Total phenolic content of *N. tabacum* extracts.

Extracts	Total phenolic content (mg gallic acid/g extract)
VL-E	59.3 ± 2.2^a^
VL-P	2.6 ± 0.6^d^
TL-E	38.0 ± 2.0^b^
TL-P	7.9 ± 0.6^c^

*Note*. G, gram; mg, milligram; TL-E, Turkish leaf ethanolic extract; TL-P, Turkish leaf petroleum ether extract; VL-E, Virginia leaf ethanolic extract; VL-P, Virginia leaf petroleum ether extract.

**Table 4:** Antimicrobial activity of *N. tabacum* extracts obtained using the disc diffusion assay.

Samples	Inhibition zone (mm)			
	*S. aureus*	*S. epidermidis*	*P. acnes*	*P. aeruginosa*
VL-E	14.00 ± 0.00^*f*^	12.00 ± 0.00^*e*^	12.47 ± 0.15^*d*^	14.23 ± 0.21^*c*^
VL-P	15.00 ± 0.00^*e*^	13.33 ± 0.23^*d*^	13.53 ± 0.15^*c*^	14.53 ± 0.15^*c*^
TL-E	16.00 ± 0.00^*d*^	13.73 ± 0.12 ^*c*^	10.57 ± 0.21^*e*^	14.53 ± 0.15^*c*^
TL-P	16.40 ± 0.00^*c*^	12.00 ± 0.00^*e*^	12.43 ± 0.12^*d*^	12.60 ± 0.10^*d*^
Ethanol	8.00 ± 0.00^g^	7.00 ± 0.00^*f*^	7.00 ± 0.00^*f*^	7.00 ± 0.00^*e*^
Petroleum ether	NI	NI	NI	NI
Ampicillin (25 *μ*g/mL)	20.80 ± 0.00^*b*^	19.63 ± 0.15^*b*^	20.67 ± 0.15^*b*^	20.27 ± 0.06^*b*^
Penicillin (25 *μ*g/mL)	28.60 ± 0.00^*a*^	25.30 ± 0.10^*a*^	25.77 ± 0.15^*a*^	26.20 ± 0.17^*a*^

*Note*. Mm, millimeter; NI, no inhibition zone; TL-E, Turkish leaf ethanolic extract; TL-P, Turkish leaf petroleum ether extract; VL-E, Virginia leaf ethanolic extract; VL-P, Virginia leaf petroleum ether extract.

**Table 5:** Antimicrobial activity of *N. tabacum* extracts obtained using the disc diffusion assay.

Samples	MIC (*μ*g/mL)			
	*S. aureus*	*S. epidermidis*	*P. acnes*	*P. aeruginosa*
VL-E	≥250	≥250	≥500	≥125
VL-P	≥125	≥250	≥250	≥125
TL-E	≥31.25	≥250	≥500	≥125
TL-P	≥15.62	≥250	≥250	≥250
Ethanol	≥1 : 2	≥1 : 2	≥1 : 2	≥1 : 2
Petroleum ether	NI	NI	NI	NI
Ampicillin (25 *μ*g/mL)	≥1.56	≥12.5	≥12.5	≥12.5
Penicillin (25 *μ*g/mL)	≥1.56	≥12.5	≥12.5	≥12.5

*Note*. MIC, minimal inhibitory concentrations; NI, no inhibition zone; TL-E, Turkish leaf ethanolic extract; TL-P, Turkish leaf petroleum ether extract; VL-E, Virginia leaf ethanolic extract; VL-P, Virginia leaf petroleum ether extract.

**Table 6:** Antimicrobial activity of *Nicotiana tabacum* extracts obtained using the minimal bactericidal concentration (MBC) method.

Samples	MBC (*μ*g/mL)			
	*S. aureus*	*S. epidermidis*	*P. acnes*	*P. aeruginosa*
VL-E	≥500	≥500	≥500	≥250
VL-P	≥125	≥250	≥250	≥125
TL-E	≥31.25	≥250	≥500	≥250
TL-P	≥15.62	≥250	≥250	≥500
Ethanol	≥1 : 4	≥1 : 2	≥1 : 2	≥1 : 4
Petroleum ether	NI	NI	NI	NI
Ampicillin 25 *μ*g/mL	≥1.56	≥12.5	≥12.5	≥12.5
Penicillin 25 *μ*g/mL	≥1.56	≥12.5	≥12.5	≥12.5

*Note*. MBC, minimal bactericidal concentrations; NI, no inhibition zone; TL-E, Turkish leaf ethanolic extract; TL-P, Turkish leaf petroleum ether extract; VL-E, Virginia leaf ethanolic extract; VL-P, Virginia leaf petroleum ether extract.

## Data Availability

The datasets used and/or analyzed during the current study can be obtained from the corresponding author upon reasonable request.
